The article "Influence of Gastrectomy on Cortical and Cancellous Bones in Rats" was retracted in 2020. Reasons: errors in the text; duplicated data; false authorship; concerns about the citations.

# Influence of Gastrectomy on Cortical and Cancellous Bones in Rats

**DOI:** 10.1155/2013/381616

**Published:** 2013-05-28

**Authors:** Jun Iwamoto, Yoshihiro Sato, Hideo Matsumoto

**Affiliations:** ^1^Institute for Integrated Sports Medicine, Keio University School of Medicine, 35 Shinanomachi, Shinjuku-ku, Tokyo 160-8582, Japan; ^2^Department of Neurology, Mitate Hospital, Fukuoka 826-0041, Japan

## Abstract

The aim of the present study was to examine the influence of gastrectomy (GX) on cortical and cancellous bones in rats. Twenty male Sprague-Dawley rats were randomized into the two groups of 10 animals each: a sham operation (control) group and a GX group. Seven weeks after surgery, the bone mineral content and density (BMC and BMD, resp.) and the mechanical strength of the femur were determined, and bone histomorphometric analyses were performed on the tibia. GX induced decreases in the BMC, BMD, ultimate force, work to failure, and stiffness of the femoral distal metaphysis and the BMC, BMD, and ultimate force of the femoral diaphysis. GX induced a decrease in cancellous bone mass, characterized by an increased osteoid thickness, osteoid surface, osteoid volume, and bone formation. GX also induced a decrease in cortical bone mass, characterized by increased endocortical bone resorption. The GX induced reductions in the bone mass and strength parameters were greater in cancellous bone than in cortical bone. The present study showed that the response of bone formation, resorption, and osteoid parameters to GX and the degree of GX-induced osteopenia and the deterioration of bone strength appeared to differ between cortical and cancellous bones in rats.

## 1. Introduction

Gastric surgery is mostly needed for the treatment of gastric cancer. After gastrectomy (GX), the daily dietary intake of calcium, magnesium, phosphorus, iron, zinc, vitamin D, vitamin B_12_, and folic acid is reported to be lower than the recommendations [1–3]. In particular, GX impairs calcium and vitamin D metabolism, leading to a risk of bone disease including not only osteoporosis, but also osteomalacia or a mixed pattern of osteoporosis osteomalacia with secondary hyperparathyroidism [4–7]. The risk for vertebral and hip fractures is increased in GX patients [7–12]. However, a strategy for preventing fractures in GX patients has not yet been established. Preclinical studies using animals could be useful for identifying available interventions to prevent fractures in GX patients.

An animal model of osteopenia can be created by performing GX in rats. Total GX and resection of the acid-producing part of the stomach (fundectomy) induces gastrinemia and malnutrition [13, 14], thereby initiating osteopenia in rats [15–19]. However, although bone histomorphometry studies have demonstrated GX-induced decreases in cancellous bone volume per tissue volume and cortical bone area in rats [17, 18], the changes in bone formation, resorption, and osteoid parameters after GX have not been adequately studied. The difference in the responses of cortical and cancellous bones to GX remains to be established in rats. Understanding the differential influence of GX on cortical and cancellous bones is important for clarifying the effect of interventions on the skeleton in GX rats. The aim of the present study was to examine the influence of GX on cortical and cancellous bones in rats.

The article "Influence of Gastrectomy on Cortical and Cancellous Bones in Rats" was retracted in 2020. Reasons: errors in the text; duplicated data; false authorship; concerns about the citations.

## 2. Materials and Methods

### 2.1. Handling of Animals

Twenty male Sprague-Dawley rats (11-week old) were purchased from Charles River Japan (Kanagawa, Japan). The animals were fed a standard pellet diet containing 1.25% calcium (calcium carbonate) and 0.9% phosphorus (CRF-1; Oriental Yeast, Co., Ltd., Tokyo, Japan). The rats were housed in a local animal room at a temperature of 24°C, a humidity of  50%, and a 12 h on/off cycle for lighting. Free access to water and a pellet diet were allowed. After 1 week of adaptation to this environment, the rats (12-week old) were sorted into strata according to body weight and were then randomized using the stratified weight method into the following two groups of 10 animals each: a sham operation control (CON) group and a GX group. A total GX was performed under general anesthesia using 25–30 mg/kg of pentobarbital (Kyoritsu Seiyaku Co., Ltd., Tokyo, Japan) injected intraperitoneally together with 2%-3% isoflurane (Mylan Inc., Tokyo, Japan) delivered via a Table Top Laboratory Animal Anesthesia System (V1 Type VetEquip, Inc., CA, USA). A longitudinal incision was made on the abdomen to expose the stomach. The whole stomach was excised, and an anastomosis of the esophagus and duodenum was performed. The weight of the rats was monitored weekly, and the duration of observation was 7 weeks. This experiment was performed at the laboratory of Hamri Co., Ltd. (Ibaraki, Japan), which has been approved by the Association for the Assessment and Accreditation of Laboratory Animal Care (AAALAC) International. The experimental protocol was approved by the Institutional Animal Care and Use Committee (IACUC) of Hamri Co., Ltd. (Ibaraki, Japan).

### 2.2. Preparation of Specimens

Rats were labeled by subcutaneous injection of 10 mg/kg of calcein (Dojindo Laboratories, Kumamoto, Japan) at 7 and 3 days before death. Seven weeks after surgery, the animals were sacrificed by exsanguination under general anesthesia with 2%-3% isoflurane (Mylan Inc., Tokyo, Japan) using a Table Top Laboratory Animal Anesthesia System (V1 Type VetEquip, Inc., CA, USA). The bilateral femora and the right tibia were harvested from each animal. The length of the left femur was measured using a dial caliper, and the weight was measured using an electronic balance (A&D Company, Tokyo, Japan). Then, the femur was preserved in saline, stored in a freezer (−60°C), and processed for the mechanical strength test. The right femur and tibia were preserved in 70% ethanol and were processed for peripheral quantitative computed tomography (pQCT) and the bone histomorphometric analysis, respectively.

The article "Influence of Gastrectomy on Cortical and Cancellous Bones in Rats" was retracted in 2020. Reasons: errors in the text; duplicated data; false authorship; concerns about the citations.

### 2.3. pQCT of the Femur

The distal metaphysis and diaphysis of the femur were scanned using pQCT (XCT-Research SA+; Stratec Medizintechnik GmbH, Pforzheim, Germany) in 70% ethanol/saline. The bones were placed horizontally in a polypropylene tube and were scanned at a voxel size of 0.12 mm. The scan line was adjusted using the scout view, and sites 3 mm and 14 mm proximal to the distal growth plate were scanned. For the analysis, a threshold of 395 mg/cm^3^ in contour mode 2 was used to separate the bone tissue from the marrow in the distal metaphysis. The total bone mineral content (BMC) and bone mineral density (BMD) were evaluated. A constant threshold of 690 mg/cm^3^ in contour mode 1 was used to separate the cortical bone from the trabecular bone in the diaphysis. The cortical thickness, BMC, and BMD were evaluated.

### 2.4. Bone Histomorphometry of the Tibia

The tibia was cut into two parts (proximal metaphysis and diaphysis plus distal metaphysis) with a diamond band saw (EXAKT BS 3000; Norderstedt, Germany), and each part was stained according to the method of Villanueva [20]. After dehydration with ethanol and acetone, the bone tissue was embedded in methyl methacrylate (Wako Pure Chemical, Japan). Frontal sections of the tibial proximal metaphysis were cut at a thickness of  5 *μ*m on a microtome (Leica RM 2065; Nussloch, Germany). Cross-sections of the tibial diaphysis were obtained 4 mm proximal to the tibiofibular junction at a thickness of 20–30 *μ*m with a microgrinder (Exakt KG 4000; Norderstedt, Germany). Then, the specimens were observed under a fluorescence microscope (Zeiss Axioplan 2; Jena, Germany) coupled with a video camera (CCD Color Camera CS 5270 I; Tokyo Electronic Industry Co., Ltd., Tokyo, Japan). A bone morphometry software program (Winroof Version 3.5; Mitani Corporation, Japan) was used for the histomorphometric analysis.

The histomorphometric parameters measured for the proximal metaphysis were the total tissue volume (TV), bone volume (BV), bone surface (BS), osteoid surface (OS), osteoid volume (OV), osteoid width (O.Wi), number of osteoid width measurements (N.O.Wi), eroded surface (ES), single- and double-labeled surfaces (sLS and dLS, resp.), interlabel width, osteoblast surface (Ob.S), osteoclast surface (Oc.S), and number of osteoclasts (N.Oc). Osteoclasts were identified as cells inside the resorption lacunae on the bone surface. The data were then used to calculate the percent cancellous bone volume (BV/TV), trabecular thickness (Tb.Th), trabecular number (Tb.N), trabecular separation (Tb.Sp), osteoid thickness (O.Th), OS/BS, OV/BV, ES/BS, mineralizing surface/BS (MS/BS), mineral apposition rate (MAR), adjusted MAR (Aj.AR), bone formation rate (BFR)/BS, Ob.S/BS, Oc.S/BS, N.Oc/BS, osteoid maturation time (Omt), and mineralization lag time (Mlt) in accordance with the standard nomenclature proposed by Parfitt et al. [21] and issues in modern bone histomorphometry [22]. Cancellous bone was assessed at a site 0.5–2.0 mm proximal to the lower margin of the growth plate and 150 *μ*m deep from the endocortical surface at the proximal metaphysis, an area that consists of secondary spongiosa.

The article "Influence of Gastrectomy on Cortical and Cancellous Bones in Rats" was retracted in 2020. Reasons: errors in the text; duplicated data; false authorship; concerns about the citations.

The parameters assessed for the diaphysis were the total tissue area (Tt.Ar), marrow area (Ma.Ar), periosteal and endocortical BS (perimeter), sLS, dLS, interlabel width, and endocortical ES, in accordance with the method described by Chen et al. [23]. The endocortical OS, Oc.S, and N.Oc were also measured. Two large cavities with and without vessels, which were independent of osteocytes and lacunae [24, 25], were observed in the intracortical area of each specimen to measure the cavity area (porotic Ar). These data were then used to calculate the cortical area (Ct.Ar), the periosteal and endocortical MS/BS, MAR, and BFR/BS, and the endocortical OS/BS, ES/BS, Oc.S/BS, N.Oc/BS, and Aj.AR.

### 2.5. Mechanical Strength Test of the Femur

Each specimen was submerged for 1 hour before testing to allow temperature equilibration. The mechanical strength of the femoral diaphysis was evaluated using the three-point bending test. A load was applied to the bone midway between two supports placed 18 mm apart. The femur was positioned so that the loading point was at the center of the femoral diaphysis, and bending occurred at the medial-lateral axis. Load-displacement curves were recorded at a crosshead speed of 5 mm/min using a material-testing machine (MZ-500S; Maruto Instrument, Tokyo, Japan). The parameters analyzed were the stiffness, work to failure, and ultimate force.

Just after the three-point bending test of the femoral diaphysis, the distal metaphysis of the femur was isolated over a length of 10 mm from the joint surface of the femoral condyle. The mechanical strength of this segment was then measured using a compression test. A compressive load was applied using a rectangular parallelepiped crosshead (length, 2 cm; width, 2 cm; and height, 1 cm) on the femoral distal metaphysis from the lateral aspect to the medial aspect. The specimens were positioned so that the loading point was at the center of the femoral lateral condyle. Load-displacement curves were recorded at a crosshead speed of 5 mm/min and a compression depth of 2.5 mm using a materials-testing machine (MZ500D; Maruto). The parameters analyzed were the stiffness, work to failure, and ultimate force.

The article "Influence of Gastrectomy on Cortical and Cancellous Bones in Rats" was retracted in 2020. Reasons: errors in the text; duplicated data; false authorship; concerns about the citations.

### 2.6. Statistical Analysis

Data were expressed as the mean ± standard deviation (SD). Comparisons among the groups were performed using an unpaired *t*-test. All the statistical analyses were performed using the Stat View J-5.0 program on a Windows computer, and a *P* value < 0.05 was regarded as significant.

## 3. Results

### 3.1. Body Weight, Femoral Length, Femoral Weight, and Femoral BMC and BMD

Table 1 shows the body weight, femoral length, femoral weight, and BMC and BMD. The initial body weight did not differ significantly between the two groups. The final body weight was lower in the GX group than in the CON group. The GX did not significantly influence the femoral length. However, the GX induced decreases in the femoral weight and the BMC and BMD of the femoral diaphysis and distal metaphysis. The GX also induced a decrease in the cortical thickness of the femoral diaphysis. The mean GX-induced reductions in the BMC and BMD of the femoral diaphysis were 22.9% and 3.2%, respectively. The mean GX-induced reductions in the BMC and BMD of the femoral distal metaphysis were 33.3% and 32.4%, respectively.

### 3.2. Bone Histomorphometric Analysis of the Tibia

Figure 1 and Table 2 show the results of the bone histomorphometric analysis of the tibial proximal metaphysis. The GX induced decreases in the BV/TV and Tb.N and an increase in the Tb.Sp without significantly influencing the Tb.Th (Figure 1). The mean GX-induced reduction in the BV/TV was 48.6%. These changes were associated with increased bone formation (Ob.S/BS, MS/BS, MAR, and BFR/BS) and increased O.Th, OS/BS, OV/BV, and Mlt (Table 2). However, the GX did not significantly influence bone resorption (ES/BS, Oc.S/BS, and N.Oc/BS) or the Omt (Table 2).

Figure 2 and Table 3 show the results of the bone histomorphometric analysis of the tibial diaphysis. GX induced a decrease in the Ct.Ar and increases in the Ma.Ar and endocortical BS (Figure 2). The mean GX-induced reduction in the Ct.Ar was 16.8%. These changes were associated with increased endocortical bone resorption (ES/BS, Oc.S/BS, and N.Oc/BS) without any significant changes in endocortical bone formation (MS/BS, MAR, and BFR/BS) (Table 3). The GX did not significantly influence the Tt.Ar or the periosteal BS (Figure 2), despite the significant but modest decrease in periosteal bone formation (MAR and BFR/BS) (Table 3). The GX did not significantly influence porotic Ar or endocortical OS/BS (Table 3).

The article "Influence of Gastrectomy on Cortical and Cancellous Bones in Rats" was retracted in 2020. Reasons: errors in the text; duplicated data; false authorship; concerns about the citations.

### 3.3. Mechanical Strength of the Femur

Figure 3 shows the results of the mechanical strength test of the femur. In the femoral diaphysis, the GX induced a decrease in the ultimate force but did not cause any significant changes in the stiffness or work to failure. In the femoral distal metaphysis, the GX induced decreases in the stiffness, work to failure, and ultimate force. The mean GX-induced reduction in the ultimate force was 21.4% for the femoral diaphysis and 36.2% for the femoral distal metaphysis.

## 4. Discussion

The present study confirmed that GX induced cortical and cancellous osteopenia, leading to a deterioration in the bone strength of the metaphysis and diaphysis in the long bones of rats. The response of bone formation, resorption, and osteoid parameters to GX and the degree of GX-induced osteopenia and the deterioration of bone strength appeared to differ between cortical and cancellous bones. These results revealed the differential responses of cortical and cancellous bones to GX in rats.

GX in rats has been reported to induce osteopenia [14, 17–19, 26–30]. In the present study, GX induced decreases in the BMC, BMD, ultimate force, work to failure, and stiffness of the femoral distal metaphysis, the BMC, BMD, and ultimate force of the femoral diaphysis, and the cancelous BV/TV and Ct.Ar in the tibia. The mean GX-induced reductions in the BMC, BMD, and ultimate force were greater in the femoral distal metaphysis (33.3%, 32.4%, and 36.2%, resp.) than in the femoral diaphysis (22.9%, 3.2%, and 21.4% resp.). The mean GX-induced reduction in BV/TV was also greater than that of Ct.Ar (48.6% and 16.8%, resp.). Thus, the GX-induced osteopenia and deterioration in bone strength were more severe at skeletal sites rich in cancellous bone, compared with those rich in cortical bone. In rats, cancellous osteopenia after GX appears to be similar to that which occurs after ovariectomy although the cortical osteopenia that occurs after GX may be more severe than that occurring after ovariectomy [17–19].

Although bone histomorphometry studies have demonstrated GX-induced decreases in cancellous BV/TV and Ct.Ar in rats [17, 18], the changes in bone formation, resorption, and osteoid parameters after GX have not been adequately studied. Furthermore, cortical bone has received less attention than cancellous bone in bone histomorphometry studies. In the present study, the GX-induced decrease in cancellous BV/TV was characterized by increases in O.Th, OS/BS, OV/BV, and bone formation, without any significant alteration in bone resorption. No significant influence on Tb.Th or Omt was seen, consistent with the results of a previous study showing that GX-induced cancellous osteopenia was characterized by a normal width but a decreased maturation time of the osteoid and an increased bone formation rate in rats [14]. As to cortical bone, a GX-induced decrease in Ct.Ar was characterized by increased endocortical bone resorption without any significant alterations in endocortical bone formation and OS/BS. The Tt.Ar and periosteal BS did not change significantly, consistent with the results of previous studies [28, 31]. These results suggested that the response of bone formation, resorption, and osteoid parameters to GX appeared to differ between cortical and cancellous bones. The risk of osteomalacia in cancellous bone must be considered after GX. GX might not influence the longitudinal bone growth [30], resulting in the nonsignificant influence of GX on the femoral length.

The article "Influence of Gastrectomy on Cortical and Cancellous Bones in Rats" was retracted in 2020. Reasons: errors in the text; duplicated data; false authorship; concerns about the citations.

Gastric acid is thought to facilitate the intestinal absorption of ingested calcium by mobilizing calcium from insoluble complexes in the diet [15]. After a GX in humans, pigs, and rats, the serum gastrin level decreases, calcium absorption is impaired, the serum calcium and 25(OH)D levels decrease, and the 1,25(OH)_2_D level increases [6, 7, 32, 33]. However, we did not evaluate the serum and urinary calcium and phosphorus levels, the serum 25(OH)D, 1,25(OH)_2_D, and parathyroid hormone (PTH) levels, or bone turnover markers. The influence of GX on these biochemical parameters may be important for translating the results of our preclinical study into clinical practice. Thus, further studies are needed to address this issue.

Approximately 80–90% of BMC is comprised of calcium and phosphorus. Other dietary components, such as protein, magnesium, zinc, copper, iron, fluoride, vitamins D, A, C, and K are required for normal bone metabolism [34]. After GX, not only calcium, phosphorus, and vitamin D, but also magnesium, iron, zinc, vitamin B_12_, and folic acid become deficient [31–33]. Zinc is essential for normal development of the skeleton [35]. Magnesium, vitamin B_12_, and folic acid are related to bone quality [36, 37]. These dietary components could have played a role in the impairment of bone mass and quality in terms of bone strength in GX rats. Although gastric acid secretion and gastric acidity have been suggested to play an important role in the intestinal absorption of calcium from ingested food or calcium salts such as calcium carbonate, available evidence suggests that gastric acid secretion and gastric acidity do not normally play a role in the absorption of dietary calcium carbonate [38]. Further studies are needed to clarify the contribution of malabsorption of nutrients, trace elements, and other vitamins in GX-induced changes in bone parameters in rats.

 Therapy of GX-induced osteopenia may consist of improving impaired calcification indicated by increased osteoid parameters in cancellous bone and increasing periosteal bone formation as well as decreasing endocortical bone resorption in cortical bone. Primarily, calcium and vitamin D supplementations are required because GX impairs calcium and vitamin D metabolism. Clinical studies showed the effects of alendronate and teriparatide on BMD in patients with postgastrectomy osteoporosis [39–41]. Preclinical study demonstrated the effect of incadronate, alendronate, estrogen, and PTH on cancellous bone mass in GX rats [42, 43]. However, a strategy for the prevention of fractures in GX patient population remains to be established although bisphosphonates and teriparatide may be good candidates for therapy of GX-induced osteopenia based on the clinical data. Further studies are needed to clarify the best therapy for GX-induced osteopenia.

The article "Influence of Gastrectomy on Cortical and Cancellous Bones in Rats" was retracted in 2020. Reasons: errors in the text; duplicated data; false authorship; concerns about the citations.

## 5. Conclusions

The present study compared the influence of GX on cortical and cancellous bones in rats and found that the responses of bone formation, resorption, and osteoid parameters to GX appear to differ between cortical and cancellous bones. GX-induced reductions in BMC, BMD, and bone strength were greater at skeletal sites rich in cancellous bone than at sites rich in cortical bone, and the GX-induced decrease in bone mass was greater in cancellous bone than in cortical bone. These differential responses of cortical and cancellous bones should be taken into consideration when clarifying the effect of interventions on the skeleton in GX rats.

## Figures and Tables

**Figure 1:** Bone histomorphometric analysis of the tibial proximal metaphysis. Structural parameters of cancellous bone. Data are expressed as the mean ± SD. An unpaired *t*-test was used to compare data between the two groups. ^a^ *P* < 0.05, ^b^ *P* < 0.001, and ^c^ *P* < 0.0001 versus GX. CON: control, GX: gastrectomy.

**Figure 2:** Bone histomorphometric analysis of the tibial diaphysis. Structural parameters of cortical bone. Data are expressed as the mean ± SD. An unpaired *t*-test was used to compare data between the two groups. ^a^ *P* < 0.001  and  ^b^ *P* < 0.0001 versus GX. CON: control, GX: gastrectomy.

The article "Influence of Gastrectomy on Cortical and Cancellous Bones in Rats" was retracted in 2020. Reasons: errors in the text; duplicated data; false authorship; concerns about the citations.

**Figure 3:** Mechanical strength of the femoral diaphysis and distal metaphysis. Data are expressed as the mean ± SD. An unpaired *t*-test was used to compare data between the two groups. ^a^ *P* < 0.05,  ^b^ *P* < 0.01, ^c^ *P* < 0.001, and  ^d^ *P* < 0.0001 versus GX. CON: control, GX: gastrectomy.

**Table 1:** Body weight and femoral length, weight, and BMC and BMD.

	Control (*n* = 10)	GX (*n* = 10)	*P* value
Initial body weight (g)	390 ± 17	383 ± 14	NS
Final body weight (g)	516 ± 35	404 ± 39	<0.0001
Femoral length (mm)	39.9 ± 0.9	39.3 ± 0.9	NS
Femoral weight (g)	1.36 ± 0.09	1.21 ± 0.09	0.0001
Femoral diaphysis			
Cortical thickness (mm)	0.807 ± 0.041	0.614 ± 0.048	<0.0001
BMC (mg/mm)	10.9 ± 0.9	8.4 ± 0.6	<0.0001
BMD (mg/cm^3^)	1372 ± 14	1328 ± 17	<0.0001
Femoral distal metaphysis			
BMC (mg/mm)	13.2 ± 1.1	8.8 ± 1.1	<0.0001
BMD (mg/cm^3^)	525 ± 39	355 ± 38	<0.0001

Data are expressed as the mean ± SD. An unpaired *t*-test was used to compare data between the two groups.

GX: gastrectomy, NS: not significant.

**Table 2:** Bone histomorphometric analysis of the tibial proximal metaphysis (formative and resorptive parameters of cancellous bone).

	Control (*n* = 10)	GX (*n* = 10)	*P* value
O.Th (*μ*m)	2.85 ± 0.30	5.54 ± 1.21	<0.0001
OS/BS (%)	8.49 ± 4.04	35.39 ± 8.84	<0.0001
OV/BV (%)	0.85 ± 0.43	6.64 ± 3.12	<0.0001
Ob.S/BS (%)	4.49 ± 2.19	25.29 ± 8.05	<0.0001
MS/BS (%)	23.9 ± 6.6	40.1 ± 4.8	<0.0001
MAR (*μ*m/day)	1.80 ± 0.31	2.97 ± 0.43	<0.0001
Aj.AR (*μ*m/day)	5.70 ± 1.61	3.51 ± 0.87	<0.01
BFR/BS (*μ*m^3^/*μ*m^2^/year)	162 ± 63	436 ± 95	<0.0001
ES/BS (%)	26.9 ± 5.0	30.9 ± 5.5	NS
Oc.S/BS (%)	5.59 ± 2.47	8.27 ± 3.56	NS
N.Oc/BS (#/mm)	1.90 ± 0.81	2.63 ± 1.11	NS
Omt (day)	1.61 ± 0.25	1.91 ± 0.54	NS
Mlt (day)	0.55 ± 0.24	1.74 ± 0.93	0.001

Data are expressed as the mean ± SD. An unpaired *t*-test was used to compare data between the two groups.

GX: gastrectomy, NS: not significant.

**Table 3:** Bone histomorphometric analysis of the tibial diaphysis (formative and resorptive parameters of cortical bone).

	Control (*n* = 10)	GX (*n* = 10)	*P* value
Periosteal			
MS/BS (%)	76.6 ± 8.0	66.4 ± 15.0	NS
MAR (*μ*m/day)	1.94 ± 0.21	1.65 ± 0.16	<0.01
BFR/BS (*μ*m^3^/*μ*m^2^/year)	546 ± 98	405 ± 121	<0.05
Endocortical			
OS/BS (%)	22.3 ± 8.9	24.9 ± 10.9	NS
MS/BS (%)	25.6 ± 7.6	23.0 ± 10.3	NS
MAR (*μ*m/day)	1.70 ± 0.58	2.00 ± 0.62	NS
Aj.AR (*μ*m/day)	1.99 ± 0.57	1.99 ± 0.91	NS
BFR/BS (*μ*m^3^/*μ*m^2^/year)	165 ± 97	176 ± 127	NS
ES/BS (%)	15.5 ± 12.1	53.9 ± 8.9	<0.0001
Oc.S/BS (%)	1.61 ± 2.06	5.92 ± 2.50	0.001
N.Oc/BS (#/mm)	0.55 ± 0.71	2.03 ± 0.83	<0.001

Data are expressed as the mean ± SD. An unpaired *t*-test was used to compare data between the two groups.

The article "Influence of Gastrectomy on Cortical and Cancellous Bones in Rats" was retracted in 2020. Reasons: errors in the text; duplicated data; false authorship; concerns about the citations.

GX: gastrectomy, NS: not significant.

## References

[1] Moizé V, Andreu A, Flores L (2013). Long-term dietary intake and nutritional deficiencies following sleeve gastrectomy or Roux-En-Y gastric bypass in a mediterranean population. *Journal of the Academy of Nutrition and Dietetics*.

[2] Pech N, Meyer F, Lippert H, Manger T, Stroh C (2012). Complications and nutrient deficiencies two years after sleeve gastrectomy. *BMC Surgery*.

[3] Pech N, Meyer F, Lippert H, Manger T, Stroh C (2012). Complications, reoperations, and nutrient deficiencies two years after sleeve gastrectomy. *Journal of Obesity*.

[4] Gennari C, Martini G, Nuti R (1998). Secondary osteoporosis. *Aging*.

[5] Tovey FI, Hall ML, Ell PJ, Hobsley M (1992). A review of postgastrectomy bone disease. *Journal of Gastroenterology and Hepatology*.

[6] Davies M, Heys SE, Selby PL, Berry JL, Mawer EB (1997). Increased catabolism of 25-hydroxyvitamin D in patients with partial gastrectomy and elevated 1,25-dihydroxyvitamin D levels. Implications for metabolic bone disease. *Journal of Clinical Endocrinology and Metabolism*.

[7] Zittel TT, Zeeb B, Maier GW (1997). High prevalence of bone disorders after gastrectomy. *American Journal of Surgery*.

[8] Melton LJ, Crowson CS, Khosla S, O’Fallon WM (1999). Fracture risk after surgery for peptic ulcer disease: a population-based cohort study. *Bone*.

[9] Kanis J, Johnell O, Gullberg B (1999). Risk factors for hip fracture in men from southern europe: The MEDOS Study. *Osteoporosis International*.

[10] Mellstrom D, Johansson C, Johnell O (1993). Osteoporosis, metabolic aberrations, and increased risk for vertebral fractures after partial gastrectomy. *Calcified Tissue International*.

[11] Glatzle J, Piert M, Meile T (2005). Prevalence of vertebral alterations and the effects of calcium and vitamin D supplementation on calcium metabolism and bone mineral density after gastrectomy. *British Journal of Surgery*.

[12] Lim JS, Kim SB, Bang HY, Cheon GJ, Lee JI (2007). High prevalence of osteoporosis in patients with gastric adenocarcinoma following gastrectomy. *World Journal of Gastroenterology*.

[13] Gepp H, Koch M, Schwille PO (2000). Vagus-sparing gastric fundectomy in the rat: development of osteopenia, relationship to urinary phosphate and net acid excretion, serum gastrin and vitamin D. *Research in Experimental Medicine*.

[14] Rümenapf G, Schwille PO, Erben RG (1997). Osteopenia following total gastrectomy in the rat—state of mineral metabolism and bone histomorphometry. *European Surgical Research*.

[15] Persson P, Gagnemo-Persson R, Chen D (1993). Gastrectomy causes bone loss in the rat: is lack of gastric acid responsible?. *Scandinavian Journal of Gastroenterology*.

The article "Influence of Gastrectomy on Cortical and Cancellous Bones in Rats" was retracted in 2020. Reasons: errors in the text; duplicated data; false authorship; concerns about the citations.

[16] Surve VV, Andersson N, Alatalo S (2001). Does combined gastrectomy and ovariectomy induce greater osteopenia in young female rats than gastrectomy alone?. *Calcified Tissue International*.

[17] Surve VV, Andersson N, Lehto-Axtelius D, Håkanson R (2001). Comparison of osteopenia after gastrectomy, ovariectomy and prednisolone treatment in the young female rat. *Acta Orthopaedica Scandinavica*.

[18] Andersson N, Surve VV, Lehto-Axtelius D (2004). Pharmacological treatment of osteopenia induced by gastrectomy or ovariectomy in young female rats. *Acta Orthopaedica Scandinavica*.

[19] Andersson N, Surve VV, Lehto-Axtelius D (2002). Drug-induced prevention of gastrectomy- and ovariectomy-induced osteopaenia in the young female rat. *Journal of Endocrinology*.

[20] Villanueva AR (1974). A bone stain for osteoid seams in fresh, unembedded, mineralized bone. *Stain Technology*.

[21] Parfitt AM, Drezner MK, Glorieux FH (1987). Bone histomorphometry: standardization of nomenclature, symbols, and units. Report of the ASBMR Histomorphometry Nomenclature Committee. *Journal of Bone and Mineral Research*.

[22] Dempster DW, Compston JE, Drezner MK (2013). Standardized nomenclature, symbols, and units for bone histomorphometry: a 2012 update of the report of the ASBMR Histomorphometry Nomenclature Committee. *Journal of Bone and Mineral Research*.

[23] Chen MM, Yeh JK, Aloia JF, Tierney JM, Sprintz S (1994). Effect of treadmill exercise on tibial cortical bone in aged female rats: a histomorphometry and dual energy x-ray absorptiometry study. *Bone*.

[24] Iwamoto J, Matsumoto H, Takeda T, Sato Y, Liu X, Yeh JK (2008). Effects of vitamin K2 and risedronate on bone formation and resorption, osteocyte lacunar system, and porosity in the cortical bone of glucocorticoid-treated rats. *Calcified Tissue International*.

[25] Iwamoto J, Matsumoto H, Takeda T, Sato Y, Yeh JK (2010). Effects of vitamin K2 on cortical and cancellous bone mass, cortical osteocyte and lacunar system, and porosity in sciatic neurectomized rats. *Calcified Tissue International*.

[26] Stenström M, Olander B, Lehto-Axtelius D, Erik Madsen J, Nordsletten L, Alm Carlsson G (2000). Bone mineral density and bone structure parameters as predictors of bone strength: an analysis using computerized microtomography and gastrectomy-induced osteopenia in the rat. *Journal of Biomechanics*.

[27] Ohta A, Motohashi Y, Sakai K, Hirayama M, Adachi T, Sakuma K (1998). Dietary fructooligosaccharides increase calcium absorption and levels of mucosal calbindin-D9k in the large intestine of gastrectomized rats. *Scandinavian Journal of Gastroenterology*.

The article "Influence of Gastrectomy on Cortical and Cancellous Bones in Rats" was retracted in 2020. Reasons: errors in the text; duplicated data; false authorship; concerns about the citations.

[28] Morohashi T, Ohta A, Yamada S (2000). Dietary fructooligosaccharides prevent a reduction of cortical and trabecular bone following total gastrectomy in rats. *Japanese Journal of Pharmacology*.

[29] Lehto-Axtelius D, Stenström M, Johnell O (1998). Osteopenia after gastrectomy, fundectomy or antrectomy: an experimental study in the rat. *Regulatory Peptides*.

[30] Mühlbauer RC, Schenk RK, Chen D, Lehto-Axtelius D, Hâkanson R (1998). Morphometric analysis of gastrectomy-evoked osteopenia. *Calcified Tissue International*.

[31] Stenström M, Olander B, Carlsson CA, Carlsson GA, Håkanson R (1995). Methodologic aspects of computed microtomography to monitor the development of osteoporosis in gastrectomized rats. *Academic Radiology*.

[32] Wojtyczka A, Bergé B, Rümenapf G (1998). Gastrectomy osteopenia in the rat: the role of vitamin B12 deficiency and the type of reconstruction of the digestive tract. *Clinical Science*.

[33] Maler GW, Kreis ME, Zittel TT, Becker HD (1997). Calcium regulation and bone mass loss after total gastrectomy in pigs. *Annals of Surgery*.

[34] Ilich JZ, Kerstetter JE (2000). Nutrition in bone health revisited: a story beyond calcium. *Journal of the American College of Nutrition*.

[35] Aaseth J, Boivin G, Andersen O (2012). Osteoporosis and trace elements—an overview. *Journal of Trace Elements in Medicine and Biology*.

[36] Iwamoto J, Takeda T, Sato Y (2006). Menatetrenone (vitamin K_2_) and bone quality in the treatment of postmenopausal osteoporosis. *Nutrition Reviews*.

[37] Sato Y, Honda Y, Iwamoto J, Kanoko T, Satoh K (2005). Effect of folate and mecobalamin on hip fractures in patients with stroke: a randomized controlled trial. *Journal of the American Medical Association*.

[38] Bo-Linn GW, Davis GR, Buddru DJ, Morawsk SG, Santa Ana C, Fordtran JS (1984). An evaluation of the importance of gastric acid secretion in the absorption of dietary calcium. *The Journal of Clinical Investigation*.

[39] Iwamoto J, Uzawa M, Sato Y, Takeda T, Matsumoto H (2010). Effect of alendronate on bone mineral density and bone turnover markers in post-gastrectomy osteoporotic patients. *Journal of Bone and Mineral Metabolism*.

[40] Bacun T, Kibel A, Pavić R (2011). Impressive results of teriparatide treatment of postgastrectomy osteoporosis. *Med Glas Ljek Komore Zenicko-Doboj Kantona*.

[41] Suzuki Y, Ishibashi Y, Omura N (2005). Alendronate improves vitamin D-resistant osteopenia triggered by gastrectomy in patients with gastric cancer followed long term. *Journal of Gastrointestinal Surgery*.

[42] Suzuki Y, Fukushima S, Iwai T (2004). Bisphosphonate incadronate prevents total gastrectomy-induced osteopenia in rats. *Bone*.

The article "Influence of Gastrectomy on Cortical and Cancellous Bones in Rats" was retracted in 2020. Reasons: errors in the text; duplicated data; false authorship; concerns about the citations.

[43] Andersson N, Surve VV, Lehto-Axtelius D (2004). Pharmacological treatment of osteopenia induced by gastrectomy or ovariectomy in young female rats. *Acta Orthopaedica Scandinavica*.

